This article has been retracted.

# High-Temperature-Resistant, Clean, and Environmental-Friendly Fracturing Fluid System and Performance Evaluation of Tight Sandstone

**DOI:** 10.1155/2022/5833491

**Published:** 2022-08-03

**Authors:** Minghao Wang, Hanlie Cheng, Jianfei Wei, Ke Zhang, David Cadasse, Qiang Qin

**Affiliations:** ^1^China United Coalbed Methane Company, Shenmu, Shaanxi 719300, China; ^2^COSL-EXPRO Testing Services (Tianjin) Co., Ltd., Tianjin 300457, China; ^3^The King's School, BP1560, Bujumbura, Burundi

## Abstract

Hydraulic fracturing, as an oil-water well stimulation and injection technology, is particularly important in the production and stimulation of low-permeability oil and gas fields, and the performance of the fracturing fluid directly affects the success of the fracturing operation. Compared with traditional water-based fracturing fluids, clean fracturing fluids have the advantages of strong sand-carrying ability and easy gel breaking with no residue. Aiming at the problem of poor temperature resistance and shear resistance of the clean fracturing fluid, based on previous research, this paper selects a high-temperature-resistant clean fracturing fluid system and evaluates the performance of the system. The research results show that the system has better rheological properties, better sand-carrying performance, shorter gel-breaking time, and less damage to the reservoir.

## 1. Introduction

Fracturing technology is famous for the shale gas revolution in the United States, but as early as 1947, American Stanolind oil and gas company conducted the first hydraulic fracturing experiment in Hugoton oilfield in southwest Kansas. On March 17, 1949, Halliburton carried out the first commercial fracturing construction in Verma, Oklahoma, and Archer County, Texas. Since then, the technology has been widely adopted by exploration and production companies around the world to improve or extend the production capacity of oil wells [1, 2]. At present, there are nearly 2.5 million fracturing operations worldwide. China began to study hydraulic fracturing technology in the 1950s and began to test it in the Yanchang oil mine in 1952. In 1973, Daqing Oilfield began to use hydraulic fracturing as an important technical measure to increase production and injection, which has a history of 30 years. With the rise of domestic shale gas development, PetroChina, Sinopec, and CNOOC have also carried out a large number of hydraulic fracturing operations in their respective oil fields [3]. Fracturing is a reservoir reconstruction technology that uses hydraulic action to form artificial fractures in oil and gas reservoirs and improve the fluid flow capacity in oil and gas reservoirs. Using the surface high-pressure pump group, we inject large displacement and high-viscosity liquid into the formation through the wellbore, and hold up the high pressure at the bottom of the well [4]. When the pressure exceeds the bearing capacity of the formation, cracks will be formed in the formation near the bottom of the well. We continuously inject the liquid-carrying proppant, and the fracture gradually extends forward. The proppant plays the role of supporting the fracture, forming a sand-filled fracture with a certain size and high conductivity so that oil and gas can easily flow into the well through the fracture, so as to achieve the effect of increasing production and injection [5, 6].

Hydraulic fracturing is an important means of developing low-pressure and permeable oil reservoirs [7, 8]. Using ground fracturing pumping equipment and its supporting sand mixer, the fracturing fluid is pumped into the fracturing target layer, pressing open the oil and gas layer, and forming one or several high-efficiency diversion fractures in the target oil and gas layer. Through fracturing construction, the fracturing fluid with a certain viscosity will greatly improve the fracturing construction efficiency, reduce the fluid loss to the formation, produce wider fractures and a good sand-carrying effect, and reduce the technological risk of fracturing construction, becoming a key factor in improving the success of fracturing operations. In the fracturing process, the fracturing fluid acts as a carrier to transmit pressure and transport proppant, and its performance affects the effect of the entire fracturing construction [9, 10]. With the improvement of fracturing technology requirements and the deepening of oil and gas reservoir exploration and exploitation, the use of the traditional water-based fracturing fluid can no longer meet the requirements.

The fracturing fluid is the working fluid of fracturing construction. It is a fluid with a certain viscosity, which plays the role of transferring energy, forming and extending fractures, and carrying proppant. At present, there are many kinds of fracturing fluids used at home and abroad, mainly oil-based fracturing fluid, water-based fracturing fluid, acid-based fracturing fluid, emulsion fracturing fluid, and foam fracturing fluid [11, 12]. Among them, the water-based fracturing fluid and oil-based fracturing fluid are widely used until today due to their advantages of low cost and convenient fluid preparation. Although hydraulic fracturing technology is an important technical guarantee for the stable production of oil and gas resources, it is widely used all over the world. However, “every coin has two sides,” so it is hydraulic fracturing [13, 14]. Hydraulic fracturing pollutes groundwater and affects human survival and development, such as spontaneous combustion of tap water. In addition, the destruction of underground rock strata by hydraulic fracturing activities may also lead to small microearthquakes. The ideal water-based fracturing fluid should have sufficient viscosity to carry proppant, and flow back quickly after fracturing, leaving no residue in the fracture and harming the formation [15]. The clean fracturing fluid is a new type of the polymer-free water-based fracturing fluid whose main component is viscoelastic surfactant, so it is also called the viscoelastic surfactant fracturing fluid. Clean fracturing fluid systems all contain one or several surfactants, which are used as thickeners in fracturing fluids due to their viscoelastic properties [16]. The clean fracturing fluid system usually includes the cationic surfactant fracturing fluid, anionic surfactant fracturing fluid, amphoteric surfactant fracturing fluid, and non-ionic surfactant fracturing fluid.

The water-based fracturing fluid system usually contains water-insoluble substances such as polymers [16]. After the gel is broken, the water-insoluble substances in the system cannot be discharged, and the remaining residues block the rock fractures and pores, seriously reducing the formation permeability and causing secondary pollution to the formation [17, 18]. The clean fracturing fluid uses viscoelastic surfactants as thickeners, and through the synergistic action of additives such as inorganic salts, the surfactant molecules are assembled into worm-like micelles in the brine solution, and the micelles are highly entangled with each other to form a three-dimensional network, resulting in viscoelasticity so that it can meet the sand-carrying requirements without cross-linking agents [19, 20]. Compared with traditional water-based fracturing fluids, clean fracturing fluids have many advantages. It has unique rheology and low viscosity, which can effectively transport proppant. It can adjust and control the filtration. Higher viscosity can be achieved at lower dosage. It is easy to prepare, simple to construct, and easy to dissolve, and does not need too much equipment. It has no polymer, is environment-friendly, exhibits good compatibility, and has no residue, no formation damage, and high pumpability [21]. With less consumption, small friction, and strong sand-carrying capacity, the oil well has increased production significantly. It has no cross-linking agent, gel breaker, and other chemical additives, and no formation damage, and can keep the filling layer in good condition [22, 23]. In this paper, a high-temperature-resistant quaternary ammonium salt clean fracturing fluid system was synthesized, and the performance of the synthesized high-temperature-resistant quaternary ammonium salt clean fracturing fluid system was evaluated by laboratory experiments, including rheology, gel breaking, sand carrying, and core damage.

## 2. Materials and Methods

### 2.1. Determination of Temperature Resistance

Fracturing fluid stability includes thermal stability and shear stability. That is, the viscosity of the fracturing fluid will not decrease significantly under temperature rise and mechanical shear, which plays a key role in the success or failure of construction. The temperature resistance performance of the high-temperature and low-damage clean fracturing fluid system is tested using the HAAKE Mars III rotational rheometer manufactured by the Thermo Corporation of the United States. We set the shear rate of the rheometer to 170 s^−1^, start the test at room temperature of 25°C, control the heating rate to be 3°C/min ± 0.2°C/min, continuously heat up to 150°C, and investigate the viscosity-temperature relationship of the clean fracturing fluid system.

### 2.2. Determination of Shear Resistance

In the clean fracturing fluid system, the viscoelastic surfactant molecules are entangled to form rod-like micelles, which in turn form a spatial network structure. Due to the reversibility of the micelle formation, its apparent viscosity does not change with time, even under high shear; once the shear rate decreases, the micelles can still aggregate and rewind again, thereby restoring the viscosity of the system, which is different from traditional polymer fracturing fluids. After the traditional plant arc glue fracturing fluid is sheared, the molecular chain is permanently disconnected, and the viscosity decreases rapidly and cannot be recovered. The shear resistance of the clean fracturing fluid system with high-temperature resistance and low damage at high temperature is tested using the HAAKE Mars III rotational rheometer manufactured by the Thermo Corporation of the United States. The shear rate is set to 170 s^−1^, the temperature is set to 120°C, and the viscosity changes are observed after 60 min of constant temperature shearing.

### 2.3. Determination of Gel Breaking and Residue

#### 2.3.1. Determination of Gel-Breaking Properties

We should try to reduce the content of water-insoluble substances in the fracturing fluid and the gel-breaking ability before flowback, reduce its blocking of rock pores and sand-filling fractures, and increase the oil and gas conductivity. In the experiment, kerosene is used as the gel breaker for the clean fracturing fluid, and the effect of kerosene addition on the apparent viscosity and gel-breaking time of the clean fracturing fluid is investigated. At 25°C, kerosene is added according to the mass ratio of 3%, 7%, and 10% of the clean fracturing fluid, and the gel breaking of the clean fracturing fluid system is investigated under a constant rotational speed. We use a capillary viscometer (*p*=0.1 mm) to measure the viscosity of the gel-breaking fluid at each time until the clean fracturing fluid system completely breaks the gel (<5 MPa·s).

#### 2.3.2. Determination of Broken Gel Residue

We take two centrifuge tubes, pour the gel-breaking liquid of the clean fracturing fluid into one of the centrifuge tubes with an initial mass of *m*1, shake well, and fill the other centrifuge tube with water of the same quality. We put two centrifuge tubes into the rotor body symmetrically, cover the top of the centrifuge tube, and set the parameters. The rotation speed is set to 3000 r/min, and the rotation time is 30 minutes. We start the centrifugation and wait for the separation to end. After the centrifugation stops rotating, we open the centrifuge tube cover, take out the centrifuge tube with the gel-breaking solution, pour out its supernatant, then put the centrifuge tube into a 110°C constant temperature oven, dry it for 4-5 h, and then transfer it to a desiccator. The mass of the centrifuge tube is weighed by an electronic balance as m2, and the residue content of the clean fracturing fluid system after gel breaking can be obtained by m2–m1.

#### 2.3.3. Determination of Static Sand-Carrying Performance

One of the functions of the fracturing fluid is to transport the proppant carried by it from the wellbore to the fractures in the production layer, delay the closure of the fractures, and form a sand-filled fracture zone with high conductivity in the oil and gas layer. The sand-carrying performance of the fracturing fluid mainly depends on its viscosity. As long as the fracturing fluid has a high viscosity, sand can be suspended in it, which is very beneficial to the distribution of sand in the fracture. However, the viscosity should not be too high. If the viscosity of the fracturing fluid is too high, the height of the fracture is large, which is not conducive to the generation of wide and long fractures. It is generally considered that the viscosity of the fracturing fluid is 50∼150 MPa·s. If the settling speed of the proppant carried by the fracturing fluid is too fast during the transportation process, the phenomenon of sand plugging in the wellbore and uneven placement of proppant in the fracture will occur, which will have an adverse effect on the stimulation of hydraulic fracturing. Therefore, evaluating the sand-carrying ability of the fracturing fluid is one of the important indicators to investigate the performance of the fracturing fluid. The sand-carrying performance of the fracturing fluid can be initially determined by the static settling rate of the proppant.

In the static settlement test, due to the existence of bubbles in the fracturing fluid hindering the settlement of quartz sand, the sand ratio of 10% is difficult to submerge into the liquid surface and uneven distribution affects the test. Therefore, small steel balls are selected to replace quartz sand in the experiment. A series of comparative experiments are conducted between the fracturing fluid and the hydroxypropyl arc glue fracturing fluid with similar viscosity.

We pour the prepared high-temperature-resistant clean fracturing fluid system into a 100 ml graduated cylinder and place it in a constant temperature water bath (70°C, 80°C, and 90°C). After specifying the temperature, we measure the liquid surface height *h* of the measuring cylinder with a ruler, use a small steel ball with a diameter of 6 nuns to lightly put it on the liquid surface, press the stopwatch, record the time for the small steel ball to reach the bottom of the measuring cylinder, and use the same method to measure the settling rate.

#### 2.3.4. Determination of Core Damage

*(1) Preliminary Preparation of Flow Medium and Core.*According to the SY/T5107-2005 test standard for evaluating the damage rate of the water-based fracturing fluid to core matrix permeability, kerosene is selected as the flow medium. The kerosene needs to be refined before the experiment. The process is as follows: We take a certain amount of kerosene, add silicon powder into it, stir evenly, and soak for a period to remove impurities and free water contained in the kerosene through the adsorption of silicon powder. Then, the kerosene is filtered by the filter funnel, and the kerosene filtrate is collected and degassed by a vacuum pump for 1 hour to complete the kerosene refining. The core is made of artificial quartz sand epoxy resin-cemented core. The core diameter is 2.503–2.504 cm, the core length is 4.09 cm, and the core is saturated with refined kerosene for 1 day.

*(2) Penetration Damage Determination Steps*

  Step 1: Pour the refined kerosene and the clean fracturing fluid after gel breaking and filtration into the high-pressure container and put the saturated core into a 25 × 80 core holder. Before the experiment starts, set the parameters, including the confining pressure value of 10 MPa, constant flow value of 2.5 ml/min, and viscosity and density values of kerosene.
  Step 2: Turn on the pump to pressurize so that the refined kerosene enters the core from the opposite end of the core holder along the pipeline to implement displacement. When there is a flowing medium, at the outlet, observe the flow value. When it is close to the set flow rate of 2.5 ml/min, start to record the permeability value, that is, the permeability before damage k1. The recording method is to record once every 3 minutes until the difference between the two adjacent values does not exceed 10%.
  Step 3: Stop the pump after obtaining a stable predamage permeability k1. Close the reverse line and connect the forward line and set the viscosity and density of the gel breaker filtrate on the instrument. Turn on the pump again so that the filtrate of the gel-breaking liquid enters the core from the inlet of the positive end of the core holder. When there is broken gel filtrate at the outlet, observe the flow value. When it is close to the set flow rate of 2.5 ml/min, start recording data and time. The method of recording data is the same as that of step 2, and the stabilization time during the recording period is not less than 30 minutes.
  Step 4: Stop the pump, close the forward line, and connect the reverse line. After setting the viscosity and density of refined kerosene on the instrument, follow the same steps as in step 2. The permeability after the flooding can be recorded as k2. The entire injury process is always performed at room temperature.

## 3. Result

### 3.1. System Optimization

On the basis that the concentration of the main agent erucamide epoxy is 4%, the salicylate (SAL) in sodium salicylate is used as the counterion to investigate the different molar ratios of sodium salicylate to erucamide epoxy (1.5 : 1, 1 : 1, and 0.5 : 1) on the viscosity of the clean fracturing fluid. Each fracturing fluid is tested on a Mars III rotational rheometer, the shear rate is set to 170 s^−1^, the heating rate is controlled to be 3°C/min°± 0.2°C/min, and the temperature is continuously increased to 150°C. The test results are shown in Figure 1.

It can be seen from Figure 1 that when the molar ratio of sodium salicylate to erucamide epoxy is 0.5 : 1 and 1.5 : 1, the fracturing fluid viscosity is always low, and the viscosity cannot reach 30 MPa·s at 130°C, indicating that it cannot effectively carry sand at high temperatures. However, when the molar ratio of sodium salicylate to erucamide epoxy is 1 : 1, the temperature resistance of the fracturing fluid is greatly improved, and the viscosity is greater than 30 MPa·s at 150°C, which meets the sand-carrying requirements at high temperatures. Therefore, choosing the molar ratio of the sodium salicylate to erucamide epoxy to be 1 : 1 is the optimal amount of counterions added.

Under the condition that the molar ratio of counterion to main agent is 1 : 1, the influence of different concentrations of main agent erucamide epoxy (2.5%, 3.5%, and 4.5%) on the viscosity of the clean fracturing fluid was investigated. The test results are shown in Figure 2.

It can be seen from Figure 2 that under a certain ratio of counterions to the main agent, the viscosity of the clean fracturing fluid increases with the increase in the mass fraction of the main agent. When the temperature exceeds 110°C, the clean fracturing fluid with a main agent concentration of 4.5% shows better temperature resistance. Although increasing the concentration of the main agent can improve the temperature resistance of the fracturing fluid, from the perspective of economy and applicability, the concentration of the main agent should generally not exceed 5%. Therefore, considering the economy and temperature resistance, it is more appropriate to choose a concentration of 4.5% of the main agent. To sum up, the clean fracturing fluid obtained when the concentration of the main agent erucamide epoxy is 4% and the molar ratio of sodium salicylate to erucamide epoxy is 1 : 1 has good high-temperature resistance.

### 3.2. Evaluation of Rheological Properties

The viscosity-temperature relationship of the high-temperature clean fracturing fluid was measured using a HAAKE Mars III rotational rheometer, and the experimental results are shown in Figure 3.

It can be seen from Figure 3 that with the increase in the test temperature, the viscosity of the high-temperature clean fracturing fluid shows a trend of first increase and then decrease, which may be related to the increase in temperature and the increase in the solubility of viscoelastic surfactant in water. The fracturing fluid viscosity peaks at 60°C. The viscosity of high-temperature clean fracturing fluid at 120°C–150°C is 31 MPa·s. The high-temperature-resistant clean fracturing fluid still has a viscosity of more than 30 MPa·s at 150°C, indicating that the fracturing fluid system at high temperature meets the sand-carrying requirements.

It can be seen from Figure 3 that the initial viscosity of the high-temperature fracturing fluid system is 80 MPa·s at 120°C, and the viscosity of the system is stable at 70 MPa·s–90 MPa·s during the subsequent 60-min constant temperature process. Under the constant temperature and constant shear rate, the viscosity of the system will not decrease, indicating that the high-temperature fracturing fluid has good shear resistance at 120°C.

### 3.3. Evaluation of Static Sand-Carrying Performance

In order to evaluate the suspending ability of the high-temperature-resistant clean fracturing fluid system and the hydroxypropyl arc glue fracturing fluid to proppant, a static sand suspension performance experiment is carried out. The experimental method is that we put the high-temperature clean fracturing fluid system into a 100 ml measuring cylinder and place it in a constant temperature water bath (70°C, 80°C, and 90°C), and wait until the fracturing fluid reaches the specified temperature. We lightly place the small steel ball on the surface of the liquid, press the stopwatch, and record the time *t* when the small steel ball reaches the bottom of the measuring cylinder. For comparison, the same method was used to measure the suspending capacity of hydroxypropyl orphan fracturing fluids of similar viscosity. The experimental results are shown in Figure 4. For the same type of the fracturing fluid, with the increase in temperature, the settlement of small balls accelerates. Under the same temperature conditions, the settling rate of small steel balls in the high-temperature clean fracturing fluid is much lower than that in the hydroxypropyl arc glue fracturing fluid. When the temperature is 90°C, the settling rate of the small steel balls in the hydroxypropyl arc glue fracturing fluid is 3 times that of the high-temperature-resistant fracturing fluid system. This shows that compared with the light propyl arc glue fracturing fluid, the high-temperature-resistant clean fracturing fluid has good sand-carrying performance. The reason for this difference is the different sand-carrying mechanisms. The orphan fracturing fluid mainly relies on polymer thickening to carry sand, while the clean fracturing fluid mainly relies on the network structure of micelle entanglement to carry sand. It can also maintain good sand suspension performance under the viscosity.

### 3.4. Gel Breaking and Residue Evaluation

#### 3.4.1. Breaking Property of the Fracturing Fluid

The breaking of the conventional vegetable gum fracturing fluid or the synthetic polymer fracturing fluid is chemical destruction; that is, the polymer chain is broken by the oxidation of the breaker so that the viscosity of the solution is rapidly reduced. The clean fracturing fluid is different; it mainly breaks the gel through contact with cinnamon or the formation of water. When the clean fracturing fluid is in contact with cinnamon, the organic matter of cinnamon enters the worm-like micelle structure, and the micelle swells, which can be decomposed into many single spherical micelles.

In the experiment, kerosene was used as the gel breaker of the clean fracturing fluid, and the gel breaking of the clean fracturing fluid after adding kerosene with a mass fraction of 3%, 7%, and 10% was investigated under constant shear rate at room temperature. The gel-breaking results of the high-temperature-resistant clean fracturing fluid are shown in Figure 5.

It can be seen from Figure 5 that with the increase in kerosene dosage, the fracturing fluid gel-breaking time is shortened. When the amount of kerosene was 3%, the clean fracturing fluid system completely broke the gel after continuous stirring for 40 minutes, and the viscosity of the gel-breaking fluid was less than 5 MPa·s; when the amount of kerosene was 10%, the clean fracturing fluid system was continuously stirred for 25 minutes. The glue-breaking effect has been achieved.

#### 3.4.2. Fracturing Fluid Gel-Breaking Residue

We put the high-temperature-resistant clean fracturing fluid into the centrifuge tube, take it out for drying after high-speed centrifugation, and calculate the residue content. The results show that the gel-breaking fluid of the high-temperature-resistant clean fracturing fluid has no residue, indicating that the fracturing fluid system after gel breaking has no damage to the formation. The main component of the clean fracturing fluid is surfactant, and its molecular diameter is only 1/5000 of that of guar gum. These small organic molecules are easily soluble in water, so no residue is produced.

### 3.5. Core Damage Evaluation

After the fracturing fluid is filtered off, the filtrate enters the formation along the fracture wall. The fracturing fluid filtrate causes the expansion of the formation of water-sensitive minerals, which reduces the porosity of the reservoir rock matrix and reduces the reservoir permeability. Therefore, the measured value of the permeability damage rate of the fracturing fluid filtrate to the reservoir matrix is also an important indicator for evaluating the quality of the fracturing fluid.

As can be seen from Figure 6, the damage rate of the high-temperature fracturing fluid to cores is 16.35%, which is much lower than the 54.5% core damage rate of the hydroxypropyl guar fracturing fluid, indicating that it has less damage to the formation and has good reservoir protection.

## 4. Conclusion

1. The shear resistance of the high-temperature clean fracturing fluid system is good. In the process of the constant temperature of 120°C and shearing for 60 min, the viscosity is stable between 70 m and 90 MPa·s. Under high temperature and constant shear rate, the viscosity of the system will not decrease, indicating that the high-temperature-resistant fracturing fluid has good shear resistance performance. The high-temperature-resistant clean fracturing fluid system can automatically break the gel after encountering kerosene. With the increase in kerosene dosage, the gel-breaking time of the clean fracturing fluid is shortened. The glue-breaking fluid of the high-temperature-resistant clean fracturing fluid system has no residue.
2. The sand-carrying performance of the high-temperature clean fracturing fluid system is better than that of the hydroxypropyl guar fracturing fluid. It can be seen from static experiments that at the same temperature, the settling rate of the small steel balls in the system is much lower than that in the hydroxypropyl guar fracturing fluid. As the temperature increases, the settling rate of the small steel balls in the fracturing fluid increases. The damage rate of the fracturing fluid system to the core is 16.35%, and the damage to the reservoir is far less than that of the hydroxypropyl guar gum fracturing fluid, which has less damage to the formation and has good reservoir protection.

## Figures and Tables

**Figure 1:** Rheological curve of different mole ratios of the fracturing fluid.

**Figure 2:** Rheological curve of different surfactant concentrations of the fracturing fluid.

**Figure 3:** Viscosity data of the clean fracturing fluid at different temperatures.

**Figure 4:** Evaluation of the static sand-carrying performance. (a) Liquid column height. (b) Setting rate.

**Figure 5:** Effect of kerosene on breaker performance of the clean fracturing fluid.

**Figure 6:** Core damage data of the clean fracturing fluid and the guar fracturing fluid.

## Data Availability

The figures used to support the findings of this study are included in the article.
